# Privacy-Preserving Sports Wearable Data Fusion Framework

**DOI:** 10.1155/2022/6131971

**Published:** 2022-05-04

**Authors:** Jia Li, Jie Zhang

**Affiliations:** Zhengzhou Preschool Education College, Zhengzhou, Henan 450000, China

## Abstract

When the sports industry has access to advanced training and preparation techniques, the sports sector is entering a new era, where real-time data processing services have a crucial priority in improving physical fitness and avoiding injuries to athletes. The primary sports support methodology is based on multiple sensors, mainly wearables, often of different types and technology, which collect somatometric data in real time and are usually analyzed with deep learning technologies. And while modern athletes train and prepare intelligently using the innovative techniques of available technology, there is considerable concern about the use of personal data. There is great concern about cyberattacks and possible data leaks that could affect the sports industry and sports in general. To secure the personal data of athletes collected and analyzed by sports wearables, this paper presents a privacy-preserving sports wearable data fusion framework. This is an advanced methodology based on Lagrange's relaxation method for the problem of multiple assignments and synthesis of information by numerous sensors and the use of differential privacy to access databases with personal information, ensuring that this information will remain personal without a third entity may disclose the identity of the athlete who provided the data.

## 1. Introduction

To overcome the competition, the modern athlete must train and prepare intelligently and take advantage of innovative techniques. Its training program must be fully personalized, incorporating advanced tools of particular precision and functionality, based on the latest scientific innovations, advanced training systems, multidisciplinary medical positions, sports researchers, and people working in advanced sports [1]. The implementation of such a program includes unique tools for monitoring the athlete's health, ergonomic characteristics, and ways to manage training load and avoid injuries [2, 3].

A key innovation used by the entire sports industry is the athlete's involvement in capturing valuable information daily [4]. The time that the athlete must devote is usually identified with the hours of his daily training, and the data recorded is generally divided into three main categories [5].

1. Wellness: The athlete's well-being is recorded daily based on his answer to seven critical questions.
2. Training load: At the end of each training unit, the athlete registers the subjective sense of effort, which leads to valuable conclusions compared to the training load designed by the coach. With these data, documented indicators are calculated, such as the weekly load change, the ratio of current and chronic load, and the monotonicity index, to capture whether the athlete is in the ideal training zone, in a subtraining zone, or has entered a zone with a high risk of injury. For example, when the current and chronic load ratio is high (>1.5), the risk of injury increases, and the training load must be corrected. Also, the weekly increase in load is an essential indicator for injury prevention. A 15% increase in load compared to the previous week causes a 50% increase in the probability of injury.
3. Health: The athlete can record extraordinary changes in his health due to illness or injury. In the purely training field, the coach undertakes the detailed planning of the training, which can be individualized and adapted, by category, for athletes who are rested, injured, absent, etc. All kinds of evaluations are collected and recorded from tests such as blood, platelets, fasting glucose, iron, creatinine, total cholesterol, up to weekly vertical jump markers, maximal oxygen uptake, but also special tests such as substance abuse control, amphetamines, cocaine, cannabinoids, barbiturates, opioids (heroin, codeine, morphine), ethanol (alcohol), benzodiazepines, and evaluation of an acceptable or nonacceptable creatinine sample.

Because it is information on an identified or identifiable physical person, all of the above information constitutes personal data. It is subject to the status of personal data legislation (“data subject”) [6]. An identifiable physical person is one whose identity can be determined, directly or indirectly, through the use of an identifier such as a name, identity number, location data, online identifier, or one or more identifiable factors such as that physical person's physical, physiological, genetic, psychological, economic, cultural, or social identity [7].

Data fusion [8] of personal data from multiple sensors for the rational use of various information is a highly complex research problem without identifying an effective solution for the functional and practical expansion of advanced personal data usage applications [9]. This view is particularly noticeable because the nature of these applications is constantly changing towards more centralized and demanding applications, where the management of incoming information is not as apparent as it was in the usually single-sensory systems of the first generation of data acquisition and management applications [10, 11]. These applications are also evolving and growing in number, incorporating increasingly sensitive information, which requires more advanced security techniques [12, 13]. All of the above introduce different types and topologies of sensors, increasing the need for a common and effective intermediate level of security between sensors and applications [14, 15].

Data mining privacy preservation entails concealing output knowledge of data through various approaches when the output data are valuable and private. This is mainly accomplished by employing two techniques: input privacy, in which information is changed using multiple styles, and output privacy, in which data are transformed to conceal the rules. Privacy preservation is critical in data mining because when data are moved or communicated between different parties, it is required to offer security to that data so that other parties do not know what information is displayed between the original parties.

Managing this coming from multiple sources different from each other complementary or surplus personal information has been recognized as a significant and critical factor in the development of sport and, in general, in preserving the prestige and credibility of the sports industry. The intermediate level of security between sensors and applications is the position occupied by the proposed privacy-preserving sports wearable data fusion framework [16, 17]. The proposed methodology ensures the integrity of the data synthesis from heterogeneous sources while guaranteeing the anonymity and reliability of the data even in cases of the use of the data in question by third-party analysts.

## 2. Related Literature

Because of the expansion of wearable devices and the fact that they manage personal data [14, 18], the research community focuses on privacy-preserving frameworks, as seen in the literature shown below.

Banerjee et al. [16] investigated the appropriateness of the Health Insurance Portability, and Accountability Act (HIPAA) concerns created by wearable technology in the IoT ecosystem, identifying legislative gaps and variables that promote health data exposure. They developed a partnership-identity risk model, showed the ramifications in four distinct settings, and offered privacy protection advice. They classified industrial self-regulation from “pure” self-regulation to “mixed” self-regulation. There is no government involvement or any other stakeholder in the private regulating mechanism, public standard setting, pricing, or output setting. There is a high level of close federal monitoring. They noted that many of the issues with health data sharing would be addressed by the business itself. However, a hybrid of industry rule-making and government monitoring has the most potential for industry self-regulation.

Zarepour et al. [19] proposed a privacy-aware architecture for wearable cameras that might safeguard all sensitive topics such as persons, objects, and places. It identifies the likely sensitive issues in each picture using contextual information acquired from the wearable sensors and stored photos. Various techniques are used to identify sensitive items after detecting the surroundings and the user's behavior. The sensitive items are first placed and then obscured or erased using image editing methods. Their findings indicated that the suggested system could identify and blur sensitive objects with sufficient precision in both an interior and an outside setting.

In 2014, Safavi et al. [20] proposed a theoretical model for wearable medical systems, which included ten concepts and nine tests capable of delivering a comprehensive privacy protection bundle to wearable device users, and which could be implemented on any wearable OS. They built this framework by examining current mobile technology, which was then coupled with current security norms and assessed using strict information security principles. They have also recommended a detailed checklist that might aid both designers and manufacturers improve the quality of their products' privacy measures. Finally, they acknowledged that these frameworks would be impossible to execute without law compliance that integrates security and confidentiality with regulation.

Chen et al. [21] introduced FedHealth, a distributed transition knowledge architecture for wearable healthcare, to address the difficulties of user data being stored in isolated islands and cloud-based models failing to personalize. FedHealth is a broad and extendable system that conducts data aggregation using federated learning and then creates reasonably tailored models using transfer learning in various healthcare applications. Their tests and applications have shown that accurate and individualized healthcare may be provided without jeopardizing privacy and security. They want to expand this technique with incremental learning in the future to provide more tailored and adaptable treatment.

Psychoula et al. [17] examined privacy resilience and methods for preserving and integrating privacy into present frameworks. As customers grow more conscious of privacy threats and demand greater privacy control from service providers, the privacy environment will evolve. Frameworks that include privacy risks might affect how data are kept, processed, and shared. They argue that data collection, management, and sharing will become even more fragmented, with each service provider having to subscribe to a user's info instead of the other side around. As a result, addressing the privacy protection dilemma requires focusing on privacy knowledge and risk. Methods for understanding and learning user preferences and negotiating to satisfy their expectations should be researched. Finally, developing algorithmic privacy risk indicators can reliably determine a person's privacy risk based on data acquired and provided about the user.

Finally, Poore et al. [22] introduced the Lagrangian relaxation method that we use, stating that these techniques have proven to be particularly helpful in solving these issues to the interference level in real time, particularly for dense scenarios and numerous scans of data from various sensors. Their research introduced a new family of creative Lagrangian relaxation methods that address some of the shortcomings of prior approaches. The efficiency and efficacy of their technique class are shown by various numerical investigations.

From the above literature, we can say that privacy-preserving [23] frameworks are under the research community's focus because of the explosion of these devices and the fact that they handle personal data [16].

## 3. Methodology

Data merging occurs when data from many sources are merged to reflect a single reference point. Although it appears to be a simple goal, data merging is a complex procedure because most databases suffer from redundancy, inconsistency, and inaccuracy. To derive significant insights from the data obtained, it is necessary to consolidate all of these data sources and get a single point of reference. The requirement for database compliance with data privacy legislation had far-reaching consequences for database management methods. However, various obstacles must be overcome to ensure database compliance with data privacy rules.

Differential privacy is a technique for publicly disclosing information about a dataset by defining the patterns of groups within the dataset while maintaining the privacy of individuals. The assumption behind differential privacy is that if the effect of a single arbitrary database modification is small enough, the query result cannot be used to infer much about any one individual, hence ensuring privacy. Differential privacy can also be defined as a constraint placed on the algorithms used to publish aggregate information about a statistical database that prevents publishing private information about individual records whose data are contained in the database. For example, some government agencies use differentially private algorithms to publish demographic data or other statistical aggregates while maintaining the confidentiality of survey responses. Businesses use them to collect information about user behavior while limiting what is visible to even internal analysts.

Differential privacy is usually considered when identifying persons whose information may be saved in a database. Although it does not explicitly address issues of identification and reidentification, differentially private algorithms are expected to be immune to such attacks. A differentially secret algorithm is one in which the observer who sees the output has no way of knowing if the computation utilizes the information of a specific individual.

The proposed methodology ensures the integrity of the data synthesis from heterogeneous sources while guaranteeing the anonymity and reliability of the data even in cases of the use of the data in question by third-party analysts [12, 24].

Specifically, having the problem of data fusion from N sensors, its modeling turns into the following optimization problem [13, 25, 26]:

(1) $$\begin{array}{c} u\left(z\right)=\underset{z_{i1}i_{2}i_{3}}{\max}\sum_{i_{1}=0}^{M_{1}}\sum_{i_{2}=0}^{M_{2}}\sum_{i_{3}=0}^{M_{3}}C_{i_{1}i_{2}i_{3}}z_{i_{1}i_{2}i_{3}}, \end{array}$$

if the following restrictions apply

(2) $$\begin{array}{c} \sum_{i_{2}=0}^{M_{2}}\sum_{i_{3}=0}^{M_{3}}z_{i_{1}i_{2}i_{3}}=1,\;i_{1}=1,2,\ldots ,M_{1},\\ \sum_{i_{1}=0}^{M_{1}}\sum_{i_{3}=0}^{M_{3}}z_{i_{1}i_{2}i_{3}}=1,\;i_{2}=1,2,\ldots ,M_{2},\\ \sum_{i_{1}=0}^{M_{1}}\sum_{i_{2}=0}^{M_{2}}z_{i_{1}i_{2}i_{3}}=1,\;i_{3}=1,2,\ldots ,M_{S}. \end{array}$$

According to Lagrange's relaxation method [22], a set of constraints is subtracted and expressed with the help of Lagrange multipliers in the objective function of the above equation. The motivation for this approach is that a proper selection of Lagrange multipliers will tend to satisfy the inherent limitations typically found in a similar problem [27]. Thus, the three-dimensional assignment problem becomes a two-dimensional assignment problem [28].

We assume that we have S sets of measurements from *N*_*S*_ sensors, which monitor an athlete and detect target points. Still, the number is not necessarily equal to the number of actual targets set in training. The S-dimensional problem is presented as follows [4, 9, 15]:

(3) $$\begin{array}{c} \max\sum_{i_{1}=0}^{M_{1}}\cdots \sum_{i_{S}=0}^{M_{S}}C_{i_{1}\ldots i_{S}}z_{i_{1}\ldots i_{S}}. \end{array}$$

Given the fact that

(4) $$\begin{array}{c} \sum_{i_{2}=0}^{M_{2}}\cdots \sum_{i_{s}=0}^{M_{S}}z_{i_{1}\cdots i_{S}}=1,\;i_{1}=1,2,\ldots ,M_{1},\\ \sum_{i_{1}=0}^{M_{1}}\cdots \sum_{i_{s}=0}^{M_{S}}z_{i_{1}\cdots i_{S}}=1,\;i_{2}=1,2,\ldots ,M_{2},\\ \cdots \\ \sum_{i_{1}=0}^{M_{1}}\cdots \sum_{i_{s-1}=0}^{M_{S-1}}z_{i_{1}\cdots i_{S}}=1,\;i_{S}=1,2,\ldots ,M_{S}. \end{array}$$

The multipliers Lagrange *u*_*r*_, *r* = *S*, *S* − 1, ... ,3 and the constraints of the above equations are defined in relation to the cost function. So, the following *r* “loose” subproblem arises [29]:

(5) $$\begin{array}{c} w_{i_{1}\cdots i_{r}}^{r}=\sum_{i_{r+1}=0}^{M_{r+1}}\cdots \sum_{i_{S}=0}^{M_{S}}z_{i_{1}\ldots i_{S}}=\sum_{i_{r+1}=0}^{M_{r+1}}w_{i_{1}\cdots i_{r+1}}^{r+1},\\ d^{i_{1}\ldots i_{r}}=\underset{i_{r+1}}{\max}\cdots \underset{i_{s}}{\max}\left(c_{i_{1}\cdots i_{S}}+u_{{\left(r+1\right)}_{i_{r+1}}}\cdots +u_{S_{i_{s}}}\right)=\underset{i_{r+1}}{\max}\left(d^{r+1_{i_{1}..i_{r+1}}}+u_{{\left(r+1\right)}_{i_{r+1}}}\right). \end{array}$$

Obviously, we have

(6) $$\begin{array}{c} d_{i_{1}\cdots i_{S}}^{S}=c_{i_{1}\ldots i_{S}}. \end{array}$$

The *r* subproblem can be written as follows:

(7) $$\begin{array}{c} \underset{w_{i_{1}-i_{r}}}{\max}\sum_{i_{1}=0}^{M_{1}}\sum_{i_{2}=0}^{M_{2}}\cdots \sum_{i_{r}=0}^{M_{r}}d^{i_{i_{1}.i_{r}}}w_{i_{1}..i_{r}}^{r_{r}}-\sum_{i_{r+1}=0}^{M_{r+1}}u_{{\left(r+1\right)}_{i_{r}+1}}\cdots -\sum_{i_{s}=0}^{M_{S}}u_{S_{i_{S}}}. \end{array}$$

Given the fact that [30]

(8) $$\begin{array}{c} \sum_{i_{2}=0}^{M_{2}}\cdots \sum_{i_{s}=0}^{M_{S}}w_{i_{1}..i_{r}}^{r}=1,\;i_{1}=1,2,\ldots ,M_{1},\\ \sum_{i_{1}=0}^{M_{1}}\cdots \sum_{i_{s}=0}^{M_{S}}w_{i_{1}..i_{r}}^{r}=1,\;i_{2}=1,2,\ldots ,M_{2}\\ ,\\ \sum_{i_{1}=0}^{M_{1}}\cdots \sum_{i_{r-1}=0}^{M_{S-1}}w_{i_{1}..i_{r}}^{r}=1,\;i_{r}=1,2,\ldots ,M_{r}. \end{array}$$

So for a given set of Lagrange multipliers, the *r* subproblem is a generalized assignment problem, where *r* *≤* *S*. We defined the binary problem because Lagrange multipliers will impose a kind of “punishment” on the relaxed constraints violated by the solution.

Because anonymizing the data set several times is not enough to protect the data from a solid and well-prepared attacker, for example, in an n-element database, a specific feature knower of n−1 objects can easily infer the value of the individual attribute that remains, and in this research, we use differential privacy, which is an interactive method that protects data, even from attackers with prior knowledge of it [31].

Given *e* > 0, a randomized function *M* yields e-differential privacy, if for every data set *x*, *x*′ with *x* ∼ *x*′ and every S ⊆ RM, where RM is the set of values of *M* [32, 33].

(9) $$\begin{array}{c} P\left[M\left(x\right)\in S\right]\leq e^{\varepsilon }\cdot P\left[M\left(x{\;}^{\prime }\right)\in S\right]. \end{array}$$

As *e* we consider a small, not negligible, positive number, usually in the interval (0.01, ln2), the lower the price, the greater the protection of records. The definition ceases to be useful if *e* < 1/*n*. We also consider *n* as universally known information. We observe that the relation can be written equivalently as follows:

(10) $$\begin{array}{c} P\left[M\left(x{\;}^{\prime }\right)\in S\right]\leq e^{\varepsilon }\cdot P\left[M\left(x\right)\in S\right], \end{array}$$

due to the symmetry resulting from the definition of the proximity of the bases. The concept of differential privacy assures us that the attacker cannot deduce from the image of *M*, most likely, if the data from a single record have changed. In some cases, it is helpful to consider a generalization of the definition.

(11) $$\begin{array}{c} P\left[M\left(x\right)\in S\right]\leq e^{\varepsilon }\cdot P\left[M\left(x{\;}^{\prime }\right)\in S\right]+\delta . \end{array}$$

The higher the *d* > 0, the easier it is for an attacker to distinguish which base is *x*′ and *x*. The initial definition (with *d* = 0) is safer. In short, term *d* represents the possibility that some people may lose more privacy than others and that the multiplication barrier does not apply to everyone. If *d* is too small, this risk is too small [34]. An overview of how differential privacy is used is shown in Figure 1.

In general, it is true that even a mechanism M : *X* - ⟶ B provides *e*-differential privacy. Then, for each function *f*, the composition *f* ◦ *M* maintains *e*-differential privacy. And this is true whether we have a sequential or adaptive composition as they will maintain (*ε*_1_ + *ε*_2_)-differential privacy. Even in the case of advanced composition, for each *ε*, *δ*, *δ*′ ≥ 0, the mechanism created by the adaptive synthesis of *k* mechanisms with (*ε*, *δ*)-differential privacy provides (*ε*′, k*δ* + *δ*′)-differential privacy with

(12) $$\begin{array}{c} \varepsilon^{\prime }=\sqrt{2k\;\log\left(\frac{1}{\delta {\;}^{\prime }}\right)}\varepsilon +k\varepsilon \left(e^{\varepsilon }-1\right). \end{array}$$

The above synthesis theorems cover both the repetitive application of differential privacy mechanisms in the same database and their repetitive application in different databases that may, however, contain information related to a specific record.

## 4. Use Case

For the modeling of the proposed system, a specialized differential privacy scenario was implemented with data derived from sensor fusion. It should be emphasized that the architecture of the models managing the randomization mechanisms is entirely different from that of the generalization mechanisms. Most algorithms use the technique to accept a set of data and return an anonymized version of it. However, the use of interactive techniques requires different modeling, and, for a question posed by a third party in the athlete's information fusion database, the administrator chooses the amount of privacy they wish to convey. The data are processed, noise is added, and the analyzer returns the result.

In the following modeling, we mainly use the Laplace mechanism, which satisfies a dynamic differential privacy criterion to implement different levels of privacy in the information distributed to third parties [35].

Let *q* be a set of values *R*, and let ∆ be its l_1_-sensitivity. Then, the mechanism [20, 33]

(13) $$\begin{array}{c} M\left(x\right)=q\left(x\right)+z, \end{array}$$

with *z* ∼ Lap(∆|*ε*), provides *e*-differential privacy.

The size of the noise depends on the type of query and the selection of *e*. So for a counting query we want order noise ∼ Lap(1|e), while the smaller the value of *ε*, the more inaccurate the result. We introduce the x-database with the athlete's heart rate and query the average heart rate [36].

(14) $$\begin{array}{c} q\left(x\right)=\frac{\sum_{i=1}^{n}x_{i}}{n}, \end{array}$$

with *x*_i_ ∈ [0, *x*_max_]. If we use a neighborhood relation of type |*x*_*i*_ − *x*_*i*_′| ≤ *x*_max_, then the sensitivity of the query will be

(15) $$\begin{array}{c} \Delta =\underset{x∼x^{\prime }}{\max}\left|q\left(x\right)-q\left(x\prime \right)\right|=\frac{1}{n}\underset{x_{i},x_{i}^{\prime }}{\max}\left|x_{i}-x_{i}^{\prime }\right|i\in \left[1,n\right]. \end{array}$$

So we have

(16) $$\begin{array}{c} \Delta =\frac{x_{\max}}{n}. \end{array}$$

According to the above, the mechanism becomes

(17) $$\begin{array}{c} M\left(x\right)=\frac{\sum_{i=1}^{n}x_{i}}{n}+\text{Lap}\left(\frac{x_{\max}}{n\varepsilon }\right), \end{array}$$

and will maintain e-differential privacy. We observe that the magnitude of the noise resulting from the Laplace mechanism is inversely proportional to the number *n* of recordings, which is to be expected since, intuitively, we expect better privacy if the size of the base is large.

The probability density function for mean µ = 0 is

(18) $$\begin{array}{c} f\left(x|0,b\right)=\frac{1}{2b}e^{-\left|x\right|/b}. \end{array}$$

So we have the cumulative distribution function

(19) $$\begin{array}{c} F\left(x\right)=\int_{-\infty }^{x}f\left(u\right)\text{d}u,\\ =\int_{-\infty }^{x}\frac{1}{2b}e^{-\left|u\right|/b}\text{d}u,\\ =\left\{\begin{array}{cc} \frac{1}{2}e^{x/b}, & x<0,\\ 1-\frac{1}{2}e^{-x/b}, & x\geq 0. \end{array}\right) \end{array}$$

The inverse function is

(20) $$\begin{array}{c} F^{-1}\left(x\right)=\left\{\begin{array}{cc} b\cdot \;\ln\left(2x\right), & 0<x<\frac{1}{2},\\ -b\cdot \;\ln\left(2-2x\right), & \frac{1}{2}\leq x\leq 1. \end{array}\right) \end{array}$$

Setting *u* = *x* - 1/2, we end up with a generator of random variables [32].

(21) $$\begin{array}{c} X=-b\cdot \mathrm{sgn}\left(u\right)\ln\left(1-2\left|u\right|\right)u\in \left(-\frac{1}{2},\frac{1}{2}\right]. \end{array}$$

Thus, by selecting random variables *u* from the uniform distribution in the interval [−0.5, 0.5], the random variable *X* will belong to the Laplace distribution with scale parameter *b*. We construct two different functions. The relation that connects *e* with the parameter *b* is

(22) $$\begin{array}{c} b=\frac{\Delta f}{\varepsilon }, \end{array}$$

with ∆f denoting the sensitivity of a function *f* : *X*⟶*ℝ*^*k*^.

(23) $$\begin{array}{c} \Delta f=\underset{x∼x{\;}^{\prime }}{\max}f\left(x\right)-f\left(x{\;}^{\prime }\right), \end{array}$$

where *x*, *x*′ are two adjacent databases.

To prove the above, we apply the proposed framework to the classic query experiment to find the mean value of a sensitive, numerical attribute. Specifically, we present in detail the methodology for finding the mean value of the heartbeat feature.

The heartbeat can be an indication of a person's physical condition. The average resting heart rate is between 70 and 75 beats per minute. People who do regular aerobic exercise reach 50 to 60 beats per minute. Professional athletes can have only 30 to 35 beats per minute, while people with poor fitness can go 90 or 100 beats per minute.

So we will have

(24) $$\begin{array}{c} f\left(x\right)=\frac{1}{n}\sum_{i=1}^{n}b_{i}. \end{array}$$

Athlete A's score values range from [30, *b*_max_]. We notice that

(25) $$\begin{array}{c} \left|b_{i}-b_{i}^{\prime }\right|\leq b_{\max}-30. \end{array}$$

Therefore, the sensitivity can be calculated as follows:

(26) $$\begin{array}{c} \Delta_{f}=\underset{x∼x{\;}^{\prime }}{\max}\left|q\left(x\right)-q\left(x{\;}^{\prime }\right)\right|=\frac{1}{n}\underset{x_{i},x_{i}^{\prime }}{\max}\left|b_{i}-b_{i}^{\prime }\right|i\in \left[1,n\right]. \end{array}$$

So we have

(27) $$\begin{array}{c} \Delta_{f}=\frac{b_{\max}-30}{n}. \end{array}$$

We know that the mechanism

(28) $$\begin{array}{c} M\left(x\right)=\frac{\sum_{i=1}^{n}b_{i}}{n}+\text{Lap}\left(\frac{b_{\max}-5}{n\varepsilon }\right), \end{array}$$

will maintain *e*-differential privacy. Applying the formula to our calculations, we get the results for the average grade.

When *e* = 1, the average grade = 33.74; when *e* = 0.1, the average grade = 33.73; and when *e* = 00.1, the average grade = 33.81, etc.

Another option is to add Laplace noise to each point and then calculate their average value.

## 5. Conclusions

To secure athletes' data collected and analyzed by sports wearables, this paper presents an innovative and highly flexible privacy-preserving sports wearable data fusion framework. It is an advanced methodology for protecting privacy in synthesized databases. Specifically, the procedure is based on the Lagrange relaxation method for the problem of multiple assignments and the synthesis of information from numerous sensors. Data are secured using a flexible, adaptive differential privacy system. Using Laplace noise allows access to databases with personal information, ensuring that this information will remain personal without a third party being able to reveal the identity of the athlete who provided the data in question.

This technique is an initial privacy-preserving framework for maintaining data mining confidentiality. When data are transferred or shared between different parties, it is mandatory to provide security so that other parties do not know what information is being shared between the original parts, identifying the users. In general, this methodology helps hide the knowledge of sports data output as the output data are valuable and private, thus contributing to the shielding of defense mechanisms related to the sports industry.

## Figures and Tables

**Figure 1:** Differential privacy (probability density vs. differential privacy output).

## Data Availability

The data used in this study are available from the corresponding author upon request.

## References

[1] Ma B., Nie S., Ji M., Song J., Wang W. (2020). Research and analysis of sports training real-time monitoring system based on mobile artificial intelligence terminal. *Wireless Communications and Mobile Computing*.

[2] Lu C. Design of information system using visual studio for auxiliary sports under computer big data.

[3] Qin G., Ding N., Yan J. Research on the intelligent system of computer big data technology to guide athletes.

[4] Patel D., Shah D., Shah M. (2020). The intertwine of brain and body: a quantitative analysis on how big data influences the system of sports. *Annals of Data Science*.

[5] Aira T., Salin K., Vasankari T. (2019). Training volume and intensity of physical activity among young athletes: the health promoting sports club (HPSC) study. *Advances in Physical Education*.

[6] Jiang R. Application of computer sports big data informatization construction comprehensive intelligent information system.

[7] Granacher U., Borde R. (2017). Effects of sport-specific training during the early stages of long-term athlete development on physical fitness, body composition, cognitive, and academic performances. *Frontiers in Physiology*.

[8] Zheng Y. (2015). Methodologies for cross-domain data fusion: an overview. *IEEE Transactions on Big Data*.

[9] El-Din D. M., Hassanien A. E., Hassanien E. E., Hassanien A. E., Bhatnagar R., Khalifa N. E. M., Taha M. H. N. (2020). Information integrity for multi-sensors data fusion in smart mobility. *Toward Social Internet of Things (SIoT): Enabling Technologies, Architectures and Applications*.

[10] Jia L., Wang Q. Establishment and application of comprehensive evaluation model for athletes.

[11] Ning X. Research and design of smart scoring system using cloud computing and big data analysis.

[12] Chen G. Research on unstructured mega data analysis algorithm of communication network based on feature fusion.

[13] Chu P., Dong Z., Chen Y., Yu C., Huang Y. Research on multi-source data fusion and mining based on big data.

[14] Wang T. Research on enterprise economic risk forecast model based on big data fusion.

[15] Nandni S., Subashree R., Tamilselvan T., Vinodhini E., Anandakumar H. A study on cognitive social data fusion.

[16] Banerjee S., Hemphill T., Longstreet P. (2018). Wearable devices and healthcare: data sharing and privacy. *The Information Society*.

[17] Psychoula I., Chen L., Amft O. (2020). Privacy risk awareness in wearables and the internet of things. *IEEE Pervasive Computing*.

[18] Lv Z., Deng W., Zhang Z., Guo N., Yan G. A data fusion and data cleaning system for smart grids big data.

[19] Zarepour E., Hosseini M., Kanhere S. S., Sowmya A. A context-based privacy preserving framework for wearable visual lifeloggers.

[20] Safavi S., Shukur Z. (2014). Conceptual privacy framework for health information on wearable device. *PLoS One*.

[21] Chen Y., Qin X., Wang J., Yu C., Gao W. (2020). FedHealth: a federated transfer learning framework for wearable healthcare. *IEEE Intelligent Systems*.

[22] Poore A. B., Robertson III A. J. (1997). A new Lagrangian relaxation based algorithm for a class of multidimensional assignment problems. *Computational Optimization and Applications*.

[23] Bringer J., Chabanne H., Patey A. (2013). Privacy-preserving biometric identification using secure multiparty computation: an overview and recent trends. *IEEE Signal Processing Magazine*.

[24] Coster D., de Witt S., Klampanos I. Towards making fusion data FAIR.

[25] Alzubaidi L., Zhang J., Humaidi A. J. (2021). Review of deep learning: concepts, CNN architectures, challenges, applications, future directions. *Journal of Big Data*.

[26] Cuzzocrea A. Big data lakes: models, frameworks, and techniques.

[27] Deb S., Yeddanapudi M., Pattipati K., Bar-Shalom Y. (1997). A generalized S-D assignment algorithm for multisensor-multitarget state estimation. *IEEE Transactions on Aerospace and Electronic Systems*.

[28] Tian N., Zhang Z. G. (2006). *Vacation Queueing Models: Theory and Applications*.

[29] Poore A. B., Gadaleta S. (2006). Some assignment problems arising from multiple target tracking. *Mathematical and Computer Modelling*.

[30] Sangüesa C. (2008). Error bounds in approximations of random sums using gamma-type operators. *Insurance: Mathematics and Economics*.

[31] Niu X., Ye Q., Zhang Y., Ye D. (2018). A privacy-preserving identification mechanism for mobile sensing systems. *IEEE Access*.

[32] D’Acquisto G., Domingo-Ferrer J., Kikiras P., Torra V., de Montjoye Y.-A., Bourka A. (2015). Privacy by design in big data: an overview of privacy enhancing technologies in the era of big data analytics. https://arxiv.org/abs/1512.06000.

[33] Hou R., Tang F., Liang S., Ling G. (2021). Multi-party verifiable privacy-preserving federated k-means clustering in outsourced environment. *Security and Communication Networks*.

[34] Cha H. J., Ahn M. L. (2014). Development of design guidelines for tools to promote differentiated instruction in classroom teaching. *Asia Pacific Education Review*.

[35] Pearn W. L., Lin P. C., Chang Y. C., Wu C.-W. (2006). Quality yield measure for processes with asymmetric tolerances. *IIE Transactions*.

[36] Torra V., Torra V. (2017). Selection of masking methods. *Data Privacy: Foundations, New Developments and the Big Data Challenge*.

